RETRACTED

# LncRNA SNHG19 Promotes the Development of Non-Small Cell Lung Cancer *via* Mediating miR-137/E2F7 Axis

**DOI:** 10.3389/fonc.2021.630241

**Published:** 2021-03-25

**Authors:** Guang-Yin Zhao, Zhao-Feng Ning, Rui Wang

**Affiliations:** ^1^ Department of Thoracic Surgery, Ruijin Hospital, Shanghai Jiaotong University School of Medicine, Shanghai, China; ^2^ Radiotherapy Branch, Cancer Hospital, Taian, China; ^3^ Department of Thoracic Surgery, The Third Affiliated Hospital of Chongqing Medical University, Chongqing, China

**Keywords:** non-small cell lung cancer (NSCLC), long non-coding RNA (LncRNA) SNHG19, MiR-137, E2F7, tumorigenesis

## Abstract

**Objective:**

Non-small cell lung cancer (NSCLC) is a common malignant tumor, which has high incidence and low the 5-year survival rate. Long non-coding RNAs (lncRNAs) play critical roles in carcinoma occurrence and metastasis. Herein, our aim was to investigate the effects of lncRNA SNHG19 in NSCLC progression.

**Materials and Methods:**

Long non-coding RNA Small Nucleolar RNA Host Gene 19 (lncRNA SNHG19) expression level was measured by bioinformatics and qRT-PCR. Edu, Transwell, and scratch assays were performed to explore the role of si-SNHG19 or SNHG19 on NSCLC progression. Luciferase assay was used to verify the relationship between SNHG19/E2F7 and miR-137. The experiment of Xenograft was used for exploring the function of SNHG19 *in vivo*.

**Results:**

SNHG19 was upregulated in cancer tissues, patients plasma and cell lines of NSCLC. Knockdown of SNHG19 inhibited cell proliferation, migration, and invasion. Luciferase assay confirmed that SNHG19 regulated E2F7 expression *via* interacting with miR-137. Overexpression of SNHG19 accelerated NSCLC tumor progression *via* miR-137/E2F7 axis both *in vitro* and *in vivo*.

**Conclusions:**

Our results clarified the SNHG19 function for the first time, and SNHG19 promoted the progression of NSCLC, which was mediated by the miR-137/E2F7 axis. This study might provide new understanding and targets for NSCLC diagnosis and treatment.

## Introduction 

Among all the malignant tumors, the incidence of lung cancer ranks first, and the incidence of lung cancer in China has been increasing for many years (1). Although medical workers have made unremitting efforts for many years, the overall 5-year survival rate of patients with lung cancer is still very low (2). Lung cancer causes more deaths than breast, colorectal, and prostate cancer combined. Non-small cell lung cancer (NSCLC) accounts for about 85% of lung cancer patients (3). About 75% of the newly treated patients with lung cancer are in the middle and late stage of inoperation. For these patients, although a variety of treatment schemes such as targeted therapy and immunotherapy have been developed in recent years, the emergence of drug resistance has seriously hindered the effect of treatment (4). It has become an important reason to limit the rehabilitation of patients in clinic.

RETRACTED

Recently, many studies have found that long non-coding RNA (lncRNA) plays an important regulatory role in the occurrence and development of tumors (5). LncRNA refers to a large class of long-stranded RNA molecules that do not encode proteins and have transcripts of more than 200 bp, which were first discovered by researchers in 2002 during the large-scale sequencing of mouse genome-wide cDNA libraries (6). Some studies have found that many lncRNAs are abnormally expressed in hepatocellular carcinoma, colorectal cancer, chronic lymphoblastic leukemia, and other malignant tumors (7, 8). In recent years, lncRNA has received more and more attention in regulating the occurrence and development of lung cancer (9). LncRNA is closely related to lung cancer, and it plays a key role in promoting the invasion and metastasis of lung cancer, promoting the growth and colony formation of NSCLC, regulating the activation of oncogenes, enhancing the stability of lung cancer cells, causing chemotherapy and targeted drug resistance (10, 11).

MicroRNA (miRNA) is an endogenous regulatory molecule, which is a small single-stranded molecule with about 21–23 bases (12). MiRNA is conserved in the process of biological evolution, through complementary binding of two nucleic acid sequences to some specific mRNA, degradation of target mRNA or inhibition of its expression at the post-transcriptional or protein translation level (13, 14). At present, a large number of studies have shown that microRNA plays an important role in the process of embryonic development and tumor occurrence and development (15). Other studies have shown that the expression pattern of miRNAs in the lung changes from fetus to adult, from normal to lung cancer; specific miRNAs may play multiple functions in the formation of the lung, and abnormal expression of miRNAs may also induce the occurrence of lung cancer (16). The imbalance between lncRNA and miRNA can lead to further deterioration of canceration of the body. Liu et al. have demonstrated that lncRNA HOTAIR is highly expressed in cervical cancer cells (17). Knockdown can inhibit the proliferation and promote apoptosis of cervical cancer cells, while miR-143-3p is lowly expressed in cervical cancer. With the decrease of miR-143-3p expression, the inhibitory effect of HOTAIR knockdown on the growth of cervical cancer cells is eliminated. Luciferase reporter gene assay confirmed that miR-143-3p was the target gene of HOTAIR. MiRNA and lncRNA can regulate each other with multiple targets, and the interaction and mode between them can be regulated by adjusting their relative abundance (18, 19). LncRNA has the recognition unit of miRNA, which can recognize miRNA, and act as a part of the miRNA interaction network, so it becomes the key regulation link of the interaction. The joint detection of miRNA and lncRNA, in tumor interaction to clarify their interaction mechanism may provide new evidence for tumor diagnosis and provide more targets for tumor treatment (20).

RETRACTED

Long non-coding RNA Small Nucleolar RNA Host Gene 19 (lncRNA SNHG19) was first identified in brain tissues of Alzheimer’s disease (21), and followed study indicated that SNHG19 was highly expressed in breast cancer tissues (22). However, the function of SNHG19 in NSCLC is poorly understood.

## Methods

### Patients’ Experiments

The surgical specimens of 60 NSCLC patients were collected from our hospital, which were used for follow-up experimental detection. 5 ml blood from 60 NSCLC patients and 20 healthy volunteers was also collected. The experiment was permitted by the Ethics Review Committee of the Third Affiliated Hospital of Chongqing Medical University, and the patients signed informed consent. Our study was conducted in accordance with the Declaration of Helsinki.

### Animal Experiments

H1650 cells of each group were prepared for inoculation for subculture for 15 generations, and the concentration was adjusted to 5 × 10^7^/0.1 ml/site and then divided into different packs. The cell suspension is blown away. Eighteen BALB/C female nude mice (4–5 weeks, weight around 20 g) were selected and grouped and numbered. Each nude mouse was weighed. The right armpit was disinfected with 75% alcohol, and 0.1 ml cell suspension was injected at each site; LCM was injected to reduce leakage and contamination. Then, lentivirus packaged SNHG19/si-SNHG19 or NC was injected through the tail vein. After inoculation, the mice were observed daily. After 4 weeks, the nude mice were collected and killed by excessive carbon dioxide, the tumors were removed, and the tumors were photographed, weighed, and recorded after all the surrounding connective tissue was removed. Tumor volume (mm3): V (Mm3) = S2 (Mm2) × L (Mm)/2. All animal experiments were performed in compliance with institutional guidelines, the National Institutes of Health guide for the care and use of Laboratory animals (NIH Publications No. 8023, revised 1978), and had been approved by Institutional Animal Care and Use Committee of the Third Affiliated Hospital of Chongqing Medical University, and the experiments were carried out following the Guide for the Care and Use of Experimental Animals.

RETRACTED

### Cell Culture and Transfection

The commonly used BEAS-2B and A549, NCI-H1299 and H1650 cell lines of NSCLC were purchased from ATCC cell center of the United States. The cells were cultured in DMEM medium with 10% fetal bovine serum and 1% dual-antibody solution in an incubator at 37°C and 5% CO_2_. The culture medium was changed every day and passed every 3 days. 500 μM miRNA or 2 μg plasmid or 2 μg siRNA was transfected into cells, which was mediated by LipofectamineTM 2000 (Invitrogen, Carlsbad, CA, USA). And plasmid or miRNA or small interfering RNA (si-RNA) was constructed and purchased from Ribobio company (Guangzhou, China).

### qRT-PCR

We used trizol method to extract total RNA from tissues, cells and peripheral blood, and RNA concentration and purity were determined using NanoDrop 2000 (Thermo Scientific, USA). RNA is used as transcription template to reverse transcribe into cDNA. Then SYBR Premix Ex TaqII was selected for RT PCR reaction. The expression value of the normal group was set as 1, and the relative expression of the experimental group was expressed as 2^−△△CT^. GAPDH was used as internal control for testing SNHG19 and E2F7, and U6 was used as control for detecting miR-137.

### Western Blot

The tissue or treated cells were lysed with lysis buffer for 30 min. After centrifugation, the supernatant was separated and placed in a 0.5 ml centrifuge tube. BCA method was used to determine the concentration of each sample, and protein loading treatment and quantitative protein samples were used. The samples were electrophoresed with polyacrylamide gel and then transferred to PVDF membrane. The PVDF membrane carrying protein was sealed with 1%BSA for 2 h and incubated with primary antibody at 4°C overnight. The second antibody was incubated the next day, and the amount of protein samples on the PVDF membrane was detected by chemical radiography. Primary antibodies list: E2F7 (ab56022, Abcam), GADPH (ab181602, Abcam).

### MTT Assay

MTT assay was used to determine the proliferative ability of cells. 100 μl (1 × 10^4^ cells) was inoculated in 96-well plates and cultured at 37°C with 5% CO_2_ for 24 h. At 24 h after transfection, 50 μl MTT solution (5 mg/ml) was added to each well, and the supernatant was discarded after incubation for 4 h at 37°C. The reduction reaction was terminated by adding 150 μl dimethyl sulfoxide (DMSO) to each well. The 96-well plate was continuously shaken for 30 min, and the optical density value of each well at 570 nm wavelength was determined, and the average value of each group was taken.

### EdU Assay

Cells at logarithmic growth stage were taken and seeded in 96-well plates with 4 × 10^3^–1×10^5^ cells per well. The cells were cultured to the normal growth stage. Transfection was performed according to experimental requirements. An appropriate amount of 50 μM Edu culture medium (Ribobio, Guangzhou) was prepared by diluting Edu solution 1,000:1. The cells were incubated at 20 μM Edu for 12 h. The cells were then fixed with 4% paraformaldehyde, stained with DAPI for 5 min, and cell proliferation was recorded by taking photos with a microscope.

RETRACTED

### Cell Migration Assay

The A549/H1650 cells were cultured in a 6-well culture plate, and after 24 h of growth at a density, they should achieve a monolayer fusion of about 70–80%. A single layer was then gently and slowly scraped with the tip of a new 200 μl pipette through the center of the hole. After scraping, the hole was gently washed twice with medium to remove the isolated cells. The cells were cultured in a fresh serum-free medium. Cell migration was recorded at 0, 24, and 48 h after culture.

### Cell Invasion Assay

The matrix glue and basic medium 1640 were fully mixed according to 1:3. A mixture of 50 μl matrix glue and basal medium 1640 was added to the bottom of the chamber. The culture plates with small Chambers were placed in a 5% CO_2_ incubator for 30 min. Single-cell suspension was prepared, and the cell concentration was adjusted to l × 10^5^/ml. In the 24-well plate, a small chamber with and without coated matrix glue was set, and a complete medium containing 10% serum was added. Cell suspension of 200 μl was slowly added into a small chamber and cultured at 37°C and 5% CO_2_ for 24 h. The cells in the small chamber were removed with a wet cotton swab and fixed immediately with formaldehyde for 5 min. After that, the small chamber was taken out and dried. Crystal violet was used for dyeing for 20 min. Then, the chamber was rinsed with water and dried. The number of transmembrane cells was observed and counted under the microscope.

### Luciferase Assay

HEK293 cells were co-transfected with 20 mmol/L miR-137 mimic or miR-NC together with wild type SNHG19 (WT-SNHG19)/mutant SNHG19 (Mut-SNHG19) or WT-E2F7/Mut-E2F7. Luciferase activity was measured with Dual Luciferase Reporter Assay Kit (Transgene, China) on GloMax20/20 at 48 h after the transfection.

### RNA-Binding Protein Immunoprecipitation

We performed a RIP assay to determine the binding between SNHG19 and miR-137 using Magna RIP™ RNA-Binding Protein Immunoprecipitation Kit (Millipore) as in a previous study (23). Briefly, A549 cells were transfected with biotinylated miR-137 or miR-NC, and the expression of SNHG19 was detected using qRT-PCR.

RETRACTED

### Ki67 Staining

Paraffin sections of carcinoma were dewaxed to water in xylene and descending series of ethanol. We penetrated sections using 0.5% Triton X-100. After washing three times, we blocked sections with 50% goat serum. Then, sections were incubated with Ki67 antibody (ab15580, Abcam) overnight. We incubated the sections using secondary antibody. The sections were photographed by light scope under an IX73 fluorescence microscope (Olympus, Valley, PA) and analyzed by Image J software.

### Statistical Analysis

Data were shown as mean ± SD. Student’s t-test or one-way ANOVA was used to compare the groups. P <0.05 was considered significant. All experiments were repeated three times.

## Results

### The Expression of lncRNA SNHG19 in NSCLC

Gene microarray was performed to identify the differentially expressed lncRNAs in normal and cancer tissues of NSCLC, which showed an increase of SNHG19 in NSCLC tissues (**Figure 1A**). Then qRT-PCR also indicated that SNHG19 was upregulated in both cancer tissues and plasma of NSCLC patients (**Figures 1B, C** **)**. Moreover, SNHG19 levels in normal (BEAS-2B) and NSCLC cell lines (A549, NCI-H1299 and H1650) were examined, and SNHG19 increased in NSCLC cell lines (**Figure 1D**).

**Figure 1:** The expression of lncRNA SNHG19 in NSCLC tissues and cells. **(A)** LncRNA expression profiles in adjacent normal tissues and cancer tissues of NCSLC patients. **(B)** We collected 60 samples of patients diagnosed with NSCLC. The expression of SNHG19 in normal and cancer tissues was detected by qRT-PCR. n = 60. **(C)** RNA in plasma of healthy volunteers and NSCLC patients was isolated, and SNHG19 expression was calculated. **(D)** qRT-PCR analysis for SNHG19 level in NSCLC cell lines (A549, NCI-H1299 and H1650) and human normal pulmonary epithelial cells BEAS-2B. Data are mean ± SD; *P < 0.05. All experiments were repeated three times.

### Silencing SNHG19 Inhibited NSCLC Growth *In Vitro*

Considering that SNHG19 had the highest expression in A549 cells, we constructed three siRNA of SNHG19 (si-NC was used as a negative control) to silence SNHG19 in A549 cells, qRT-PCR assay was used to detect the inhibition efficiency (**Figure 2A**). 2^#^ si-SNHG19 was selected for subsequent functional experiments. MTT assay indicated that deletion of SNHG19 inhibited cell viability (**Figure 2B**). Edu analysis indicated that deletion of SNHG19 inhibited proliferative viability (**Figure 2C**). Scratch test showed that si-SNHG19 suppressed cell migrate rate (**Figure 2D**). Besides, transwell assay exhibited that si-SNHG19 reduced invasive ability of A549 cells (**Figure 2E**).

**Figure 2:** Deletion of SNHG19 inhibited the proliferation, migration and invasion of A549 cells. Small interfering RNA of SNHG19 (si-SNHG19) and its NC (si-NC) were transfected into A549 cells. **(A)** The knockdown efficiency of si-SNHG19 was determined by qRT-PCR. **(B)** MTT assay used to detect cell viability. **(C)** EdU assay was to detected proliferation of A549 cells. Scale bar, 20 μm. **(D)** Wound healing assay was to evaluate migration of A549 cells. Scale bar, 100 μm. **(E)** Transwell assay was to examine invasion of A549 cells. Scale bar, 50 μm. Data are mean ± SD; *P < 0.05. All experiments were repeated three times. ns, no significant.

RETRACTED

### SNHG19 Interacted With miR-137 and Regulated E2F7 Expression in NSCLC Cells

At present, it has been found that lncRNA regulates miRNA by acting as the precursor of miRNA, competitively combining mRNA with miRNA and “sponge effect” (24). Through the prediction of the bioinformatics website (Lncbook, DIANA, Starbase), we found that miR-137 may be a target of lncRNA SNHG19 (**Figure 3A**). The binding site was predicted, and luciferase assay reported that miR-137 could combine with WT-SNHG19, but not with Mut-SNHG19 (**Figure 3B**). Moreover, RIP assay showed an increasing enrichment of SNHG19 in bio-miR-137 group than in bio-miR-NC group (**Figure 3C**). After transfection with sh-SNHG19/sh-NC in A549 cells, the expression of miR-137 was increased in the sh-SNHG19 group (**Figure 3D**), and the expression of SNHG19 was decreased after miR-137 mimic transfection (**Figure 3E** **)**. In NSCLC cell lines and patient’s tissues, the level of miR-137 was significantly reduced (**Figures 3F, G** **)**. In addition, miR-137 was downregulated in NSCLC patient’s plasma (**Figure 3H**). Correlation analysis using ENCORI website showed that there was a negative correlation between SNHG19 and miR-137 in lung adenocarcinoma (LUAD) (**Figure 3I**). As shown in **Figure 3J**, E2F7 might be a potential target of miR-137. Luciferase assay reported that miR-137 could interact with E2F7 (**Figure 3K**). The expression level of E2F7 was decreased in A549 cells after sh-SNHG19 transfection, while SNHG19 promoted E2F7 expression (**Figure 3L**). And E2F7 was highly expressed in NCSLC tissues than that in normal tissues (**Figure 3M**). Taken together, SNHG19 could regulate E2F7 level *via* sponging miR-137.

**Figure 3:** SNHG19 acted as a sponge of miR-137 and modulated E2F7 expression. **(A)** Bioinformatics used to predict the targets of SNHG19, which showed that miR-137 may be a target of lncRNA SNHG19. **(B)** The binding sites between SNHG19 and miR-137 were shown. Wild type and mutant SNHG19 was transfected into HEK293 cells with or without miR-137, and luciferase assay was to evaluate the binding between miR-137 and SNHG19. **(C)** RIP used to determine the binding between SNHG19 and miR-137 in A549 cells. **(D)** A549 cells were transfected with SNHG19 plasmid or si-SNHG19 or its NC, the mRNA level of miR-137 was detected using qRT-PCR. **(E)** A549 cells were transfected with miR-137/miR-NC, and SNHG19 expression was tested. The level of miR-137 in NSCLC cell lines **(F)**, patient’s tissues **(G)** and plasma **(H)** was detected. **(I)** ENCORI website used to determine the correlation between SNHG19 and miR-137 in lung adenocarcinoma (LUAD). **(J)** Bioinformatics used to predict the targets of miR-137. **(K)** The binding sites between E2F7 and miR-137 were shown. Wild type and mutant E2F7 was transfected into HEK293 cells with or without miR-137, and luciferase activity was tested. **(L)** A549 cells were transfected with SNHG19 plasmid or si-SNHG19 or its NC, the protein level of E2F7 was detected using western blot. **(M)** E2F7 expression in normal and cancerous tissues was detected. Data are mean ± SD; *P < 0.05, ns, no statistical significance. All experiments were repeated three times.

RETRACTED

### SNHG19 Promoted Growth *via* miR-137/E2F7 Axis in NSCLC Cells

We then detected the role of miR-137 in the progression of NSCLC cells. A549 cells were transfected with miR-137 mimics or miR-NC, and the expression of miR-137 in A549 cell was increased (**Supplementary Figure 1A**). Following functional experiments indicated that overexpression of miR-137 inhibited cell proliferation, migration, and invasion in A549 cells (**Supplementary Figures 1B, C** **)**. Because SNHG19 had the lowest expression in H1650 cells, we forced expression of SNHG19 with miR-137 mimics or si-E2F7 in H1650 cells (**Figure 4A**). SNHG19 promoted cell proliferation, migration, and invasion in H1650 cells (**Figures 4B–E**). However, miR-137 mimics or si-E2F7 removed the promoting role of SNHG19 on NSCLC cells (**Figures 4B–E**). Moreover, considering the differential expression of SNHG19/miR-137/E2F7 axis in plasma of NSCLC patients, ENCORI database was used to determine the role of SNHG19/miR-137/E2F7 axis in lung cancer patients’ survival. And we found that high expression of SNHG19 and low expression of miR-137 indicated a lower survival rate, and high expression of E2F7 indicated a lower survival rate (**Supplementary Figures 2A–C**).

**Figure 4:** SNHG19 promoted NSCLC growth through miR-137/E2F7 axis. SNHG19 was transfected into H1650 cells with miR-137 or si-E2F7. **(A)** The transfection efficiency was detected using qRT-PCR. **(B)** MTT analysis for cell viability of H1650 cells. **(C)** Edu assay for cell proliferation of H1650 cells. Scale bar, 20 μm. **(D)** Wound healing assay for cell migration of H1650 cells. Scale bar, 100 μm. **(E)** Transwell assay for cell invasion of H1650 cells. Scale bar, 50 μm. Data are mean ± SD; *P < 0.05 *vs* pcDNA3.1, ^#^P < 0.05 *vs* SNHG19. All experiments were repeated three times.

RETRACTED

### SNHG19 Promoted NSCLC Tumorigenesis *In Vivo*

We implemented tumor formation in nude mice. H1650 cells were subcutaneously injected into the right lower limb of the nude mice; then lentivirus packaged SNHG19 was injected through the tail vein. SNHG19 enhanced the tumor volume (**Figure 5A**), and increased the ratio of tumor weight to body weight (**Figure 5B**). In addition, isolated tumor tissues had a higher SNHG19 level after injection (**Figure 5C**). Moreover, injection of SNHG19 reduced the mRNA level of miR-137, and induced E2F7 expression (**Figures 5D, E** **)**. Ki67 staining indicated that SNHG19 induced the expression of Ki67 in isolated tumor tissues, which suggested that SNHG19 promoted tumor cell proliferation (**Figure 5F**). While inhibition of SNHG19 *in vivo* showed an opposite effect, si-SNHG19 inhibited tumor weight and tumor volume comparing with si-NC (**Supplementary Figures 3A, B** **)**. And si-SNHG19 promoted miR-137 expression and inhibited E2F7 level in isolated tumor (**Supplementary Figure 3C**).

**Figure 5:** SNHG19 promoted NSCLC growth *in vivo*. 30 mice were divided into two groups randomly, H1650 cells were subcutaneously injected into nude mice. And lentivirus packaged SNHG19 or pcDNA3.1 was injected through the tail vein. **(A)** Tumors were isolated after injection of H1650 cells. **(B)** Tumor volume was measured every 7 days. **(C)** The ratio of tumor weigh to body weight was calculated. **(D)** The mRNA of SNHG19, miR-137, and E2F7 in isolated tumors was detected by qRT-PCR. **(E)** The protein level of E2F7 in isolated tumors. **(F)** Ki67 staining was used to detect proliferation of isolated tumors. Data are mean ± SD; *P < 0.05. All experiments were repeated three times.

## Discussion

Today, as a high incidence of malignant tumor, the 5-year survival rate of NSCLC is significantly lower than that of breast cancer, prostate cancer, and other common tumors (25). The main cause of death is tumor invasion and metastasis (26). These pathophysiological changes are not only a signal of disease progression, but also the main cause of treatment failure. Although we have done a lot of research on tumor invasion and metastasis, the specific mechanism of its development is still unclear (27). At present, a large number of studies have found that the occurrence and metastasis of lung cancer are affected not only by genes, but also by external factors such as small RNA and long non-coding RNA. A lot of evidence shows that they play an important role in a variety of diseases (28).

RETRACTED

In recent years, the function of lncRNA in life activities has been continuously discovered with the extensive development of research. Through genome sequencing analysis, many lncRNAs are found to be involved in biological activities such as transcriptional activation, transcriptional interference, and chromatin modification (29). In addition, lncRNA plays an important role in the mutagenesis and metastasis of tumor cells. The expression profiles of many lncRNAs in lung cancer cells have changed significantly compared with normal cells (30). These abnormally expressed lncRNA involve a number of biological processes, including gene transcription and protein translation. Not only that, it may also involve the splicing of mRNA and the regulation of cell cycle and so on. There are many signs that they can play a role not only in the process of protein expression, but also in the process of modification after proteome expression, or in the process of protein–protein interaction (31).

At present, the specific role of SNHG19 in tumor is not clear. We found the expression of SNHG19 in lung tissue for the first time, and its expression was significantly increased in NSCLC tissue than that in normal para-carcinoma tissue. Moreover, SNHG19 was also highly expressed in plasma of patients with lung cancer. These results suggest that SNHG19 might be used as a diagnostic marker of lung cancer and played a regulatory role in the occurrence and development of NSCLC, which pushed us to further explore the function of SNHG19 in NSCLC. There is evidence that the abnormal expression of lncRNA in tumors indicates the role of promoting or inhibiting tumors. The expression of HOTAIR is increased in lung cancer tissues, and it promotes the proliferation and migration of lung cancer cells by negatively regulating the expression of miR-326 (32). Wang et al. have shown that UCA1 is highly expressed in lung cancer cells and can be used as a predictive marker of lung cancer. The upregulation of UCA1 will lead to poor clinical prognosis (33). UCA1 promotes the growth of NSCLC cells by competitively combining the expression of miR-193a-3p-targeted ERBB4 (11). The carcinogenic effect of UCA1 is related to the downregulation of miR-193a-3p expression. Inhibition of UCA1 expression can reduce the colony formation of NSCLC cells. The study also confirmed that UCA1 is related to miR-143 and regulates the expression of miR-143 target HK2, which strongly proves that UCA1 is regulating gene expression at the post-transcriptional level (34). In present, we used siRNA of SNHG19 to inhibit SNHG19 expression in NSCLC cells, which was a common method to knock down gene expression in cells. Cell proliferation is the key process for tumor growth, and cell migration and invasion contribute to proximal and distant metastases of tumor (35). Thus, we assessed NSCLC cells’ proliferation, migration, and invasion after silencing SNHG19. Interestingly, si-SNHG19 inhibited the proliferation, migration, and invasion of NSCLC cells.

RETRACTED

Many studies have pointed out that lncRNA, like mRNA, can bind with miRNA to inhibit the downregulation of mRNA expression by miRNA, thus realizing the regulatory function (24). Through the screening and comparison of multiple databases, we found that miR-137 existed in the binding site of SNHG19, and luciferase experiments proved that there was a binding relationship between them. Moreover, E2F7 was a direct target of miR-137. MiR-137 was shown to downregulate in lung cancer and involved in cell survival and proliferation (36). LncRNA XIST induced PXN expression *via* binding miR-137, which promoted cell viability and invasion in NSCLC (37). E2F7 contributes to the occurrence and development of multiple tumors, including NSCLC, prostate cancer, and colon cancer (23, 38, 39). Our study further revealed that overexpression of SNHG19 promoted NSCLC cells’ proliferation, migration, and invasion, while miR-137 or si-E2F7 remitted the motivating effect of SNHG19. Moreover, SNHG19 accelerated tumor growth *in vivo*.

## Conclusion

In summary, our results clarified the SNHG19 function for the first time, and SNHG19 promoted the progression of NSCLC, which was mediated by the miR-137/E2F7 axis. This study might provide new understanding and targets for NSCLC diagnosis and treatment.

## Data Availability Statement

The original contributions presented in the study are included in the article/**Supplementary Material**. Further inquiries can be directed to the corresponding author.

## Ethics Statement

The studies involving human participants were reviewed and approved by the Third Affiliated Hospital of Chongqing Medical University. The patients/participants provided their written informed consent to participate in this study. The animal study was reviewed and approved by Third Affiliated Hospital of Chongqing Medical University.

## Author Contributions

G-YZ and Z-FN contributed to the conception or design of the work. RW contributed to the acquisition, analysis, or interpretation of data for the work. ZN drafted the manuscript. G-YZ critically revised the manuscript. All gave final approval and agree to be accountable for all aspects of work ensuring integrity and accuracy. All authors contributed to the article and approved the submitted version.

RETRACTED

## Conflict of Interest

The authors declare that the research was conducted in the absence of any commercial or financial relationships that could be construed as a potential conflict of interest.

## Supplementary Material

Supplementary Figure 1 The role of miR-137 on the progression of A549 cells. A549 cells were transfected with miR-137 mimics or miR-NC. **(A)** miR-137 transfection efficiency was evaluated by qRT-PCR analysis. **(B)** MTT assay for cell viability. **(C)** EdU assay for proliferation of A549 cells. Scale bar, 20 μm. **(D)** Wound healing assay for migration of A549 cells. Scale bar, 100 μm. **(E)** Transwell assay for invasion of A549 cells. Scale bar, 50 μm. Data are mean ± SD; *P < 0.05. All experiments were repeated three times.

Supplementary Figure 2 ENCORI database used to determine the role of SNHG19/miR-137/E2F7 in lung cancer patients’ survival. **(A)** Lung squamous cell carcinoma (LUSC) patients with high expression of SNHG19 had a lower survival in 150 months. The effect of miR-137 **(B)** and E2F7 **(C)** in survival of lung adenocarcinoma (LUAD) patients.

Supplementary Figure 3 Inhibition of SNHG19 suppressed NSCLC growth in vivo. 30 mice were divided into two group randomly, A549 cells were subcutaneously injected into nude mice. And lentivirus packaged si-SNHG19 or si-NC was injected through tail vein. **(A)** Tumors was isolated after 4 weeks of A549 cells injection. And Tumor volume was measured every 7 days. **(B)** The ratio of tumor weigh to body weight was calculated. **(C)** The mRNA of SNHG19, miR-137, and E2F7 in isolated tumors were detected by qRT-PCR. *P < 0.05.
